The article "The Practical Effect of Action Intervention Strategy Combined Based on Surgical and Psychological Factors" was retracted in 2023. Reasons: signs of a paper mill; compromised peer review; unreliable results or conclusions.

# The Practical Effect of Action Intervention Strategy Combined Based on Surgical and Psychological Factors

**DOI:** 10.1155/2022/4591982

**Published:** 2022-10-05

**Authors:** Haiyan Tong, Jingjuan Xu, Lin Tang

**Affiliations:** ^1^Department of General Surgery, Anqing Municipal Hospital, Anqing 246003, China; ^2^School of Nursing, Soochow University, Suzhou 215006, China; ^3^Third Affiliated Hospital of Soochow University, Suzhou 215006, China; ^4^Dialysis Room, Anqing Municipal Hospital, Anqing 246003, China

## Abstract

This study mainly analyzes the related surgical and psychological factors that cause the change of thirst degree after gastrointestinal surgery, and observes the practical effect of action intervention strategy combined with the two factors on reducing postoperative thirst degree. Based on this, the clinical data of 87 patients who underwent gastrointestinal tumor resection in our hospital from January 2020 to January 2021 is retrospectively analyzed. The degree of thirst is evaluated by the visual analogue scale (VAS) and the subjects are divided into three groups: a mild group (*n* = 29), a moderate group (*n* = 35), and a severe group (*n* = 23), and their psychological and surgical indicators are compared and analyzed. The results show that the thirst degree and light comfort of mouth in the study group are better than those in the control group at 2 h after surgery, and there is no significant difference when compared to 6 h after surgery, but the thirst degree and oral discomfort in the control group at 6 h after surgery are significantly higher than those in the study group at 2 h after surgery. It is suggested that an action research intervention strategy with a high practical effect can effectively reduce postoperative thirst and oral discomfort.

## 1. Introduction

As an invasive treatment, gastrointestinal surgery mainly involves the removal of gastrointestinal tumors. In addition, perioperative fasting, water prohibition, anesthesia, mechanical ventilation, intubation, and other factors will lead to varying degrees of postoperative thirst symptoms [1]. According to clinically incomplete statistics, the majority of patients in surgical postoperative 6 h are accompanied by strong thirst symptoms, and more than 70% of patients with moderately severe thirst accounted for; patients with a serious thirst not only cause physical discomfort but may also cause psychological distress in a state of anxiety; adherence to treatment and rehabilitation progress produces serious influence [2, 3]. Therefore, as one of the main factors affecting the recovery and prognosis of the disease, thirst assessment plays an important role in alleviating the symptoms of thirst and speeding up recovery by understanding the risk factors that cause thirst and reducing postoperative thirst [4]. Therefore, in the first part of this study, the relevant factors leading to the increased thirst degree of patients after gastrointestinal surgery in our hospital are analyzed from both the surgical and psychological aspects through retrospective experiments.

The article "The Practical Effect of Action Intervention Strategy Combined Based on Surgical and Psychological Factors" was retracted in 2023. Reasons: signs of a paper mill; compromised peer review; unreliable results or conclusions.

In addition, according to the relevant expert guidelines of the department of rehabilitation, for patients with gastrointestinal motility barriers, the symptoms of thirst can be alleviated by resuming a normal diet in a short period after surgery, but a period of fasting and water restriction is still reserved for the sake of safety in clinical practice [5]. Although relevant studies have shown that postoperative stimulation of salivary gland secretion by linear tube tools can relieve patients' thirst symptoms to a certain extent, it is limited to unilateral intervention and lacks comprehensive action-based intervention measures [6, 7]. Therefore, in the second part of this study, an intervention trial is conducted to formulate corresponding strategies by combining the theory and practice of the first part and observing its practical effect in the clinical application process, so as to provide a theoretical basis for further improving the prognosis of patients after gastrointestinal surgery.

The rest of this paper is organized as follows: Section 2 discusses related work.  Section 3 is the evaluation of thirst degree and oral comfort. Analyzing the causes of thirst after gastrointestinal surgery is discussed in Section 4.  Section 5 concludes the paper with a summary.

## 2. Related Work

Thirst, as one of the most direct subjective feelings of the human body, is a sense that regulates volume and body fluid balance. There are various factors causing thirst in daily life, including frequent urination, diabetes, kidney disease, and diet. Under normal circumstances, the body's internal and external fluid cells are in a state of balance. The body by continuous vasopressin secretion and activation of the sympathetic system reduced the exclude who also solute and kidney, but for gastrointestinal surgery patients, due to the invasive operation pressure of balance resulting in serious water loss, thus the thirsty silvered tax act, which coordinated physiological balance [8]. After the operation, the gastrointestinal tract of the patient gradually disappeared with the effect of anesthesia, and various functions of the body gradually recovered. Severe thirst could cause the patient to be in a state of restlessness and lead to a series of adverse prognoses such as wound dehiscence, increased blood pressure, bleeding, and arrhythmia. Therefore, it was of great significance to understand the relevant factors that caused postoperative thirst and carry out targeted interventions to promote the recovery of patients and improve the poor prognosis [9, 10].

The article "The Practical Effect of Action Intervention Strategy Combined Based on Surgical and Psychological Factors" was retracted in 2023. Reasons: signs of a paper mill; compromised peer review; unreliable results or conclusions.

From surgery-related metrics, endotracheal intubation time, systolic pressure, diastolic blood pressure, and blood sugar levels were the causes of postoperative patients with thirst degree, aggravating the related risk factors, including the longer intubation in patients with a high degree of postoperative thirst [11]. Blood pressure level, as another risk factor affecting postoperative thirst, would compress the osmolar receptors of the internal carotid artery, resulting in increased osmolar pressure and increased thirst [12]. The higher the intraoperative blood glucose concentration, the heavier the postoperative thirst. This was mainly due to the relatively strong stress response during invasive surgery, which caused a sharp rise in glucagon, glucocorticoid, and other glucocorticoids. High blood sugar would lead to high blood sugar in the intraoperative reaction, and high blood sugar would increase blood coagulation, thereby increasing the burden of metabolism on the liver and kidney and not secreting enough albumin to store enough water, resulting in strong thirst [13].

From psychology-related metrics, depression, anxiety, and preoperative psychological elastic ability were associated with thirst postoperatively in patients with a severe degree of increasing risk factors, including depression and anxiety as a kind of negative emotion; both would speed up the body's consumption to a different degree, result in long-term strained nerve and muscle, and accelerate moisture evaporation [14]. The mental resilience ability referred to the patient's ability to adjust to different environments. Therefore, when the patient had a strong psychological ability to adjust, it could effectively relieve their own depression and anxiety before surgery [15, 16].

## 3. Evaluation of Thirst Degree and Oral Comfort

The clinical data of 87 patients who underwent gastrointestinal tumor resection at our hospital from January 2020 to January 2021 were selected for retrospective analysis. The thirst degree is evaluated by the visual analogue scale (VAS), and they are divided into three groups: a mild group (*n* = 29), a moderate group (*n* = 35), and a severe group (*n* = 23).

In the intervention study, 100 patients who undergo gastrointestinal tumor resection in our hospital from February 2021 to May 2022 are selected and divided into the study group (*n* = 50) and control group (*n* = 50) by a random number table method. All patients are put into Excel according to the code of 1–100, and even numbers are included in the study group and singular numbers in the control group. The patients included in the study all meet the relevant standards for gastrointestinal tumors and signed surgical consent before surgery. Patients with mental instability, oral disease, and contraindications are excluded.

The article "The Practical Effect of Action Intervention Strategy Combined Based on Surgical and Psychological Factors" was retracted in 2023. Reasons: signs of a paper mill; compromised peer review; unreliable results or conclusions.

The degree of thirst is evaluated by the researchers using a double-blind method. The researchers do not know the groups in advance, and the degree of thirst is objectively evaluated according to the number of thirsts, chapped lips, and thirst time interval. 4 to 6 times is reduced to 2 points, 7 to 10 times or more is recorded as 3 points, and 10 times is reduced to 4 points; no chapped lips are scored 1-point, slight peeling is scored 2 points, and severely chapped lips are scored 3 points. Thirst interval ≥5 h is 1 point, 2–4 h is 2 points, < 2 h is 3 points, and the total score is 1–10 points. The higher the score, the more thirsty you are.

Oral comfort is assessed using the VAS scoring method, with a score ranging from 0 to 10 points. Mild thirst/mild oral discomfort ≤3 points, moderate thirst/moderate oral discomfort 4–7 points. > 7 points for severe thirst/severe oral discomfort, based on the 6-hour postoperative score.

The self-rating anxiety scale (SAS) and self-rating depression scale (SDS) are used to evaluate the anxiety and depression of the patients before surgery, respectively. The two scoring scales adopt a 4-level scoring system, with branches ranging from 0 to 100, and the higher the score, the more serious the anxiety and depression.

The Connor- Davidson Resilience Scale (CD-RISC) is used to assess the patient's mental resilience before surgery. A 5-level scoring system is adopted, with 25 items and 100 points in total. The higher the score, the better the patient's mental resilience.

In the intervention experiment, an action intervention strategy is adopted for the research group. First, an action intervention group is established, mainly composed of nurses with deputy director qualifications, nurses in charge, and doctors, to collect risk factors causing postoperative thirst and coordinate the progress of each task. The action research method is used as the main framework of the intervention strategy, and the above risk factors are planned, observed, and reflected in a cyclic revision to ensure their clinical effect. Before surgery, teach patients about postoperative thirst so that patients understand that postoperative thirst is a normal phenomenon, eliminate postoperative anxiety and fear of the unknown, and guide patients to master corresponding measures when they have thirst symptoms and can operate on their own. During the operation, the patient can be timely supplemented with intravenous fluid according to the doctor's advice. After surgery, the oral cavity is moistened with a sterile elephant nose spray bottle in a reasonable way. At the same time interval, the watering can be filled with ice and salt water to gently wet the mouth.

The article "The Practical Effect of Action Intervention Strategy Combined Based on Surgical and Psychological Factors" was retracted in 2023. Reasons: signs of a paper mill; compromised peer review; unreliable results or conclusions.

SPSS 25.0 statistical software is used for data analysis. Measurement data: if the normality test conforms to a normal distribution with homogeneity of variance, it is expressed as the mean ± standard deviation. A paired sample *t*-test is used within groups; variance comparisons between groups are used; and repeated measures analysis of variance is used for comparisons between groups in each time period, and a spherical test is also used. Statistics: descriptive statistical analysis is performed using percentile and x2 tests. All the above data are significantly different, *P* < 0.05.

## 4. Analyzing the Causes of Thirst after Gastrointestinal Surgery

### 4.1. Comparison of Baseline Data between Mild, Moderate, and Severe Groups

Table 1 shows the comparison of baseline data. It is clearly evident from Table 1 that BMI is not significant.

### 4.2. Comparison of Surgical Indicators in Patients with Different Thirst Levels

Table 2 shows the comparison of surgical indicators in patients with different thirst levels. It is clearly evident from Table 2 that patients with different degrees of thirst have significant differences in endotracheal intubation time, systolic blood pressure, diastolic blood pressure, and blood glucose (*P* < 0.05).

### 4.3. Multivariate Analysis of Surgical Factors Causing Thirst after Gastrointestinal Surgery

Table 3 shows the multivariate analysis of surgical factors causing thirst after gastrointestinal tract surgery. It is clearly evident from Table 3 that the result has a significant difference among the three groups in 2.2 indicators as independent variables.

Figure 1 shows the forest regression of surgical factors. It is clearly evident from Figure 1 that endotracheal intubation time, systolic pressure, diastolic blood pressure, and blood sugar levels are the cause of postoperative patients with thirst degree, aggravating the related risk factors.

### 4.4. Psychological Indicators of Patients with Different Thirst Levels

Table 4 shows the psychological indicators of patients with different thirst levels. It is clearly evident from Table 4 that patients with different degrees of thirst have significant differences in anxiety, depression, and mental resilience.

### 4.5. Multivariate Analysis of Psychological Factors Causing Thirst after Gastrointestinal Surgery

Table 5 shows the multifactorial analysis of psychological factors causing thirst after gastrointestinal surgery. It is clearly evident from Table 5 that psychological indicators with significant differences among the three groups in 2.4 are taken as independent variables.

The article "The Practical Effect of Action Intervention Strategy Combined Based on Surgical and Psychological Factors" was retracted in 2023. Reasons: signs of a paper mill; compromised peer review; unreliable results or conclusions.

Figure 2 shows the forest regression of psychological factors. It is clearly evident from Figure 2 that anxiety, depression, and mental resilience are all related risk factors leading to increased postoperative thirst.

### 4.6. Comparison of Baseline Data between the Two Groups

Table 6 shows the comparison of baseline data. It is clearly evident from Table 6 that the comparison of baseline data between the two groups of patients grouped in the intervention test is comparable.

### 4.7. Change of Thirst at 2 h and 6 h after Operation

Table 7 shows the change in thirst at 2 h and 6 h after the operation. It is clearly evident from Table 7 that the thirst degree in the study group is significantly lower than that in the control group.

Figure 3 shows how the thirst degrees of the two groups changed at each time point after the operation. It is clearly evident from Figure 3 that although the thirst degree increases in both groups 6 h after surgery, the change in the study group is not statistically significant.

### 4.8. Oral Comfort Score of Each Group at 2 h and 6 h after Surgery

Table 8 shows the oral comfort score at 2 h and 6 h after the operation. It is clearly evident from Table 8 that 2 hours after surgery, the oral discomfort of the study group is lighter than that of the control group.

Figure 4 shows how the oral comfort of the two groups changed at each time point after the operation. It is clearly evident from Figure 4 that although there is no significant difference compared with 6 hours after surgery, the oral discomfort shows a downward trend.

## 5. Conclusion

Since the severity of thirst during the recovery of patients after gastrointestinal surgery is closely related to the prognosis, if the thirst problem of patients cannot be effectively alleviated, it will cause irritability, restlessness, and other adverse emotions, and further hinder the follow-up rehabilitation treatment and recovery speed. Surgical factors such as tracheal intubation time, systolic blood pressure, diastolic blood pressure, and blood sugar levels as well as psychological factors such as depression, anxiety, and mental flexibility are the main factors that aggravate postoperative thirst. Thirst level, improve oral comfort, with a high practical effect.

## Figures and Tables

**Figure 1:** Forest regression of surgical factors.

The article "The Practical Effect of Action Intervention Strategy Combined Based on Surgical and Psychological Factors" was retracted in 2023. Reasons: signs of a paper mill; compromised peer review; unreliable results or conclusions.

**Figure 2:** Forest regression of psychological factors.

**Figure 3:** The thirst degree of the two groups changed at each time point after the operation.

**Figure 4:** The oral comfort of the two groups changed at each time point after the operation.

**Table 1:** Comparison of baseline data.

Group	Number	Age (years)	Gender		Asa grade		BMI (kg/m^2^)
			Man	Woman	I	II	
Mild group	29	46.41 ± 8.00	15 (51.72)	14 (48.28)	17 (58.62)	12 (41.38)	24.82 ± 0.76
Moderate group	35	47.46 ± 7.37	18 (51.43)	17 (48.57)	20 (57.14)	15 (42.86)	24.41 ± 1.01
Moderate group	23	48.91 ± 6.51	13 (56.52)	10 (43.48)	16 (69.57)	7 (30.43)	24.59 ± 0.82
*F*		0.737	0.168		0.996		1.711
*P*		0.482	0.920		0.680		0.187

**Table 2:** The operative indicators of patients with different degrees of thirst.

	Mild group (*n* = 29)	Moderate group (*n* = 35)	Moderate group (*n* = 23)	*F*	*P*
Operating time (h)	2.48 ± 0.68	2.45 ± 0.65	2.54 ± 0.63	0.157	0.855
Anesthesia time (h)	3.06 ± 0.56	2.81 ± 0.63	2.90 ± 0.77	1.153	0.321
Preoperative water restriction time (h)	8.93 ± 0.68	8.63 ± 0.63	8.56 ± 0.68	2.414	0.096
Endotracheal intubation time (h)	21.14 ± 1.02	22.73 ± 0.95	26.64 ± 1.55	150.004	＜0.001
SBP (mm·HG)	123.21 ± 4.41	127.26 ± 4.35	142.48 ± 7.91	84.918	＜0.001
DBP (mm·HG)	74.24 ± 2.92	80.43 ± 3.13	88.83 ± 3.68	131.913	<0.001
Blood glucose (mmol/L)	5.61 ± 0.29	6.84 ± 0.50	8.08 ± 0.21	274.535	<0.001

**Table 3:** Multivariate analysis of surgical factors causing thirst after gastrointestinal tract surgery.

	*B*	*S.E.*	*Wald*	*P*	*OR*	*95%CI*
Endotracheal intubation time	1.035	1.121	4.857	0.002	0.142	0.085∼0.683
SBP	1.419	0.732	5.235	0.023	0.467	0.256∼0.673
DBP	3.211	1.212	3.642	0.004	0.642	0.114∼0.895
Blood glucose	1.283	0.834	3.411	0.001	0.271	0.081∼0.671

**Table 4:** The psychological indicators of patients with different thirst levels.

	Mild group (*n* = 29)	Moderate group (*n* = 35)	Moderate group (*n* = 23)	*F*	*P*
SAS	40.48 ± 5.76	61.20 ± 8.33	70.52 ± 9.19	103.841	<0.001
SDS	43.66 ± 5.33	61.14 ± 6.02	74.09 ± 8.46	142.362	<0.001
CD-RISC	81.41 ± 7.89	71.06 ± 5.67	57.78 ± 4.46	91.924	<0.001

**Table 5:** Multifactorial analysis of psychological factors causing thirst after gastrointestinal surgery.

	*B*	*S.E.*	*Wald*	*P*	*OR*	*95%CI*
SAS	1.144	1.821	4.354	0.003	0.178	0.046∼0.458
SDS	3.821	1.312	3.391	<0.001	0.632	0.152∼0.874
CD-RISC	−1.185	0.486	3.672	0.001	0.318	0.192∼0.782

**Table 6:** Comparison of baseline data.

Group	Number	Age (years)	Gender		Asa grade		BMI (kg/m^2^)
			Man	Woman	I	II	
Study group	50	46.56 ± 7.37	27 (54.00)	23 (46.00)	31 (62.00)	19 (38.00)	24.52 ± 0.88
Control group	50	47.18 ± 7.20	30 (60.00)	20 (40.00)	33 (66.00)	17 (34.00)	24.50 ± 0.90
*t*/*x*^2^		−0.426	0.367		0.174		0.097
*P*		0.671	0.545		0.677		0.923

The article "The Practical Effect of Action Intervention Strategy Combined Based on Surgical and Psychological Factors" was retracted in 2023. Reasons: signs of a paper mill; compromised peer review; unreliable results or conclusions.

**Table 7:** Changes of thirst at 2 h and 6 h after operation.

Group	Number	2 h after surgery	6 h after surgery	*t*	*P*
Study group	50	5.54 ± 1.16	5.80 ± 1.03	−1.097	0.278
Control group	50	6.54 ± 1.27	7.18 ± 1.16	−2.898	0.006
*t*		−4.113	−6.305		
*P*		＜0.001	＜0.001		

**Table 8:** Oral comfort score at 2 h and 6 h after operation.

Group	Number	2 h after surgery	6 h after surgery	*t*	*P*
Study group	50	4.44 ± 1.22	4.26 ± 1.05	0.852	0.398
Control group	50	5.90 ± 1.04	7.12 ± 1.40	−4.826	＜0.001
*t*		−6.468	−11.601		
*P*		＜0.001	＜0.001		

## Data Availability

The experimental data used to support the findings of this study are available from the corresponding author upon request.
